The article "Finite versus Indefinite Nucleos(t)ide Analogue Therapy of Patients with Chronic Hepatitis B Exhibiting Negative HBsAg Levels after Treatment" was retracted in 2024. Reasons: signs of a paper mill; suspected computer-generated content; unreliable results or conclusions; concerns about the data.

# Finite versus Indefinite Nucleos(t)ide Analogue Therapy of Patients with Chronic Hepatitis B Exhibiting Negative HBsAg Levels after Treatment

**DOI:** 10.1155/2022/6069781

**Published:** 2022-07-15

**Authors:** Haixia Sun, Yinhui Liu, Yufeng Zhang, Yusheng Jie, Yuankai Wu, Zhanyi Li, Xuxia Wei, Xiangyong Li

**Affiliations:** ^1^Department of Infectious Diseases, The Third Affiliated Hospital of Zhongshan University, No. 600 Tianhe Road, Guangzhou, 510000 Guangdong, China; ^2^Department of Infectious Diseases, People's Hospital of Foshan Sanshui District, No. 16 Southwest Guanghai Avenue West, Foshan 528100, Guangdong Province, China; ^3^Department of Surgical Intensive Care Unit, The Third Affiliated Hospital of Zhongshan University, No. 600 Tianhe Road, Guangzhou, 510000 Guangdong, China

## Abstract

**Aim:**

To determine whether a decrease in HBsAg to <0.05 IU/mL could be a criterion for cessation of finite nucleos(t)ide analogue (NUC) therapy in patients with chronic hepatitis B (CHB).

**Methods:**

This was a retrospective analysis of 6715 patients with CHB between January 1998 and May 2016. Patients were followed up every 12–24 weeks. Among 104 patients achieving HBsAg levels < 0.05 IU/mL, 71 were eligible for inclusion in the analysis: 31 received finite NUC therapy, and 40 received indefinite NUC therapy. In the finite therapy group, 9 patients received no NUC consolidation therapy, 6 received short-term (<1 year) consolidation, and 16 received long-term (>1 year) consolidation. The outcome measures were alanine aminotransferase (ALT), total bilirubin, albumin, hepatitis B virus DNA, and HBsAg levels.

**Results:**

Baseline parameters and characteristics at the time when HBsAg levels had fallen to <0.05 IU/mL were similar between the finite and indefinite therapy groups. No patients experienced viral breakthrough/relapse during a median follow-up of 120 weeks. There were little or no differences in long-term outcomes between the finite and indefinite therapy groups and between the short-term and long-term consolidation groups.

**Conclusions:**

Discontinuation of NUCs may be acceptable in patients whose HBsAg levels fall to <0.05 IU/mL. Consolidation therapy lasting <1 year appears adequate to prevent poor long-term prognosis.

## 1. Introduction

Clinical decision-making regarding the discontinuation of nucleos(t)ide analogue (NUC) therapy in patients with chronic hepatitis B (CHB) has recently become a subject of heated debate [1–3]. Conflicting factors that complicate whether to discontinue NUC therapy include the risks of viral breakthrough and relapse, hepatocellular carcinoma (HCC), liver cirrhosis, and patient preference [4, 5]. The ideal outcomes of NUC therapy are a sustained off-treatment viral response, normal alanine aminotransferase (ALT) level, and persistently reduced risk of HCC [1–3, 6, 7]. However, these outcomes are often difficult to achieve due to the stable integration of the covalently closed circular DNA into the host genome [8].

Finite therapy with NUCs is an attractive strategy because indefinite use of NUCs is limited by several factors such as the economic burden of a long treatment course, risk of nonadherence to treatment, incidence of viral breakthrough, and increasing risk of adverse effects with increasing treatment time [1–3]. Nevertheless, viral relapse and consequent exacerbation of hepatitis after cessation of NUCs are nonnegligible risks of the finite approach to treatment [9, 10]. The key requirement for finite therapy is the identification of an evidence-based marker for discontinuation. For hepatitis B e antigen- (HBeAg-) positive patients, HBeAg seroconversion was considered a potential marker for NUC discontinuation [1]. Unfortunately, several studies have demonstrated that a large proportion of patients experience viral relapse and elevations of ALT upon discontinuation of NUC treatment following HBeAg seroconversion [1, 7, 8, 11]. As an alternative criterion, loss of hepatitis B surface antigen (HBsAg) was found to be a much safer potential endpoint since NUC discontinuation after loss of HBsAg did not result in adverse events in most cases [5]. However, no studies have directly compared finite and indefinite NUC therapy for patients achieving HBsAg loss following treatment. In addition, recent technological advances now allow the detection of very low levels of HBsAg, whereas previous guidelines relied on detection thresholds that may not have reliably identified the loss of HBsAg [2–4, 6].

Prospective trials to investigate this issue are unfeasible because of the low frequency and unpredictability of the endpoints. Therefore, the present retrospective study is aimed at determining whether a decrease in HBsAg to very low levels (<0.05 IU/mL) could be used as a marker for cessation of NUC therapy by comparing the benefits and outcomes of the finite and indefinite approaches.

## 2. Methods

### 2.1. Study Design and Patients

This was a retrospective analysis of consecutive patients with CHB seen at our hospital (Guangzhou, China) between January 1998 and May 2016. This study was approved by the Clinical Ethics Review Board at our hospital. Written informed consent was obtained from all patients at the time of recruitment.

The inclusion criteria were as follows: (1) age ≥ 18 years; (2) HBsAg-positive for more than 6 months; (3) met the indications for antiviral therapy described in the guidelines for the prevention and treatment of CHB drawn up by the Chinese Society of Hepatology and the Chinese Society of Infectious Diseases (Chinese Medical Association); (4) received NUCs at our hospital according to the applicable guidelines at the time of recruitment [2–6]; and (5) HBsAg levels fell to <0.05 IU/mL (considered as HBsAg-negative) during NUC therapy. The exclusion criteria were as follows: (1) coinfection with another hepatitis virus; (2) coexistence of alcoholic, drug-induced, or autoimmune liver disease; (3) pregnant or breastfeeding woman; (4) liver cirrhosis; (5) liver cancer; (6) lost to follow-up; and (7) inadequate serum available for analysis.

### 2.2. Follow-Up

All patients were followed up at intervals of 12–24 weeks. Serum levels of hepatitis B virus (HBV) DNA, HBsAg, HBeAg, ALT, albumin, and total bilirubin were tested at each follow-up visit. The last follow-up was on 31 March 2016.

### 2.3. Data Collection

Age, gender, diagnosis of fatty liver, HBeAg status, and serum levels of ALT, albumin, total bilirubin, and HBV DNA were documented at each follow-up. Serum levels of HBV DNA, HBsAg, HBeAg, and anti-HBe were reanalyzed using serum samples stored at -80°C to avoid potential bias caused by the use of different testing techniques during follow-up. HBV DNA levels were measured using a real-time PCR assay (DAAN Gene Co., Ltd., Guangzhou, China), which had a detection threshold of 100 IU/mL. HBsAg, HBeAg, and anti-HBe were measured using commercially available chemiluminescence assay kits (Roche Diagnostics, Indianapolis, IN, USA).

### 2.4. Definitions of Treatment Approaches

Finite treatment was defined as a finite duration of NUC therapy after the patient had achieved HBsAg level < 0.05 IU/mL with or without consolidation therapy. Indefinite treatment was defined as the continuous administration of NUCs without interruption or cessation. Consolidation therapy was defined as prolonged uninterrupted administration of NUCs after the HBsAg level had fallen to <0.05 IU/mL in patients undergoing finite NUC therapy. Short-term consolidation was defined as consolidation therapy lasting <1 year, while long-term consolidation was defined as consolidation therapy for ≥1 year.

### 2.5. Outcome Measures

The outcome after discontinuation of therapy was classified as either “sustained response” or “virological relapse.” Sustained response was defined as a serological, virological, and biochemical response that was sustained after cessation of therapy [7]. Virological relapse was defined as off-therapy HBV DNA levels > 2000 IU/mL in at least two measurements performed >4 weeks apart. Virological breakthrough was defined as HBV DNA levels > 2000 IU/mL in at least two determinations performed >2 weeks apart during NUC therapy [8]. Abnormal levels of ALT, albumin, and total bilirubin were defined as levels greater than the upper limits of normal.

### 2.6. Statistical Analysis

Normally distributed continuous variables are presented as the mean ± standard deviation and were analyzed using Student's *t*-test. Nonnormally distributed variables are presented as median (range) and were analyzed using the Mann–Whitney *U* test. Categorical variables are presented as frequencies and were analyzed using the chi-squared test or Fisher's exact test, as appropriate. Statistical analysis was performed using SPSS 20.0 (IBM Corp., Armonk, NY, USA). Two-sided *P* values < 0.05 were considered statistically significant.

## 3. Results

### 3.1. Characteristics of the Patients

A total of 6715 patients were assessed for eligibility, and 104 of these achieved HBsAg < 0.05 IU/mL during treatment with NUCs. Thirty-three of these 104 patients were excluded for the following reasons: inadequate serum for analysis (*n* = 16), liver cirrhosis (*n* = 9), lost to follow-up (*n* = 5), and hepatocellular carcinoma (*n* = 3). Therefore, 71 patients were eligible for this analysis (Figure 1). Among the 71 patients included in the final analysis, 31 received finite NUC therapy (finite NUC group) and 40 received indefinite NUC therapy (indefinite NUC group).

The baseline demographic and clinical characteristics did not differ significantly between the two groups of patients, both at the time when NUC therapy was started and at the time when the HBsAg level fell to <0.05 IU/mL (Table 1). Moreover, the baseline characteristics remained unchanged when the patients in the finite NUC group discontinued NUCs after different durations of consolidation therapy (Table 2). The 71 patients included in the analysis were followed up for a median of 120 weeks (range: 24–240 weeks).

### 3.2. Indefinite NUC Therapy Did Not Improve Long-Term Outcomes Compared with Finite NUC Therapy

The long-term outcomes for finite and indefinite treatment with NUCs were compared to determine the benefits of a finite treatment approach for patients achieving very low levels of HBsAg. None of the patients in either treatment group experienced viral breakthrough/relapse once HBsAg levels had fallen below 0.05 IU/mL; only one patient in the finite NUC group exhibited a transient increase in HBsAg levels, but this was without consequence and did not require the readministration of NUCs. ALT levels were not significantly different between the two groups (Figure 2). However, patients receiving indefinite NUC therapy exhibited a higher incidence of abnormalities than those in the finite treatment group (*P* < 0.05 at the start of treatment and *P* < 0.01 after 48, 72, 96, and 120 weeks of follow-up; Figure 2). Albumin levels were slightly lower in the indefinite treatment group at 24 and 48 weeks after HBsAg had fallen to <0.05 IU/mL (*P* < 0.05; Figure 2). Total bilirubin levels showed a significant increase in the finite treatment group at 24 weeks after HBsAg had reached <0.05 IU/mL (*P* < 0.05), but overall, the total bilirubin levels and rates of abnormality were similar between the two groups (Figure 2).

To avoid bias caused by different consolidation periods, the prognoses of the patients in the finite NUC group after discontinuation of therapy were compared with the prognoses of patients in the indefinite treatment group. ALT levels, albumin levels, and the rates of abnormality in ALT and albumin levels were not significantly different between the two groups (Figure 3). Total bilirubin levels were higher in the indefinite NUC group at 24 weeks after HBsAg had reached very low levels than in the finite NUC group at 24 weeks after NUC withdrawal (*P* < 0.05), although no significant differences were observed at all other time points (Figure 3). Furthermore, both groups had similar rates of abnormality in total bilirubin level (Figure 3).

### 3.3. Baseline Characteristics of the Finite NUC Group according to the Duration of the Consolidation Therapy with NUCs

In the finite treatment group, 9 patients did not receive consolidation therapy; i.e., NUC therapy was discontinued when their HBsAg levels reached <0.05 IU/mL. Among those patients in the finite treatment group receiving consolidation with NUCs, 6 patients received short-term (<1 year) consolidation therapy while 16 patients were given long-term (≥1 year) consolidation therapy (Figure 4). Seven of the 16 patients receiving long-term consolidation therapy were given >2 years of treatment (Figure 4). Although the long-term consolidation therapy group had a lower proportion of male patients than the short-term consolidation therapy group (0.0% vs. 73.3%, *P* = 0.043), the other baseline characteristics did not differ significantly between groups both at the time when the HBsAg level reached <0.05 IU/mL and at the time of NUC discontinuation (Table 3).

### 3.4. Long-Term NUC Consolidation Therapy Does Not Improve Long-Term Outcomes Compared with Short-Term NUC Consolidation Therapy

Assessment of long-term outcomes revealed that the ALT, total bilirubin, and albumin levels were similar between the short-term consolidation therapy group and long-term consolidation therapy group (Figures 5 and 6).

## 4. Discussion

The aim of the present study was to compare finite versus indefinite NUC therapy in patients with CHB who had achieved HBsAg levels < 0.05 IU/mL following treatment. The results suggest that discontinuation of NUCs may be acceptable in patients whose HBsAg levels fall to <0.05 IU/mL. Furthermore, consolidation therapy lasting <1 year appears to be adequate in the prevention of a poor long-term prognosis.

An important finding of this study was that indefinite NUC therapy did not provide any additional benefits compared with finite NUC therapy during a median follow-up of 120 weeks. None of the patients in the finite NUC group experienced viral relapse upon discontinuation of the treatment and none required the readministration of NUCs. Since most patients in the finite NUC group received consolidation therapy of varying durations, the outcomes of the finite and indefinite treatment strategies were compared using withdrawal of the NUCs as the start of the follow-up for the finite NUC group; the results of this analysis indicated that the outcomes were similar between groups. Previous studies of the outcomes of patients with HBsAg conversion reported safety profiles that agreed with our findings [5, 12], but it must be stressed that there were several differences between the studies in terms of the study population (country, ethnicity, life habits, and healthcare system) and study design. Nevertheless, in the systematic review by Chang et al. [12], the clinical benefits and risks were found to be similar between the finite and indefinite treatment approaches, consistent with the observations of the present study. Nonetheless, defining an appropriate criterion for withdrawal of NUC therapy will be critical for the successful implementation of a finite NUC treatment strategy in clinical practice [12]. Based on the data in the present study, discontinuation of NUCs after the HBsAg level reaches <0.05 IU/mL could be an acceptable treatment strategy, especially when the nonclinical benefits of the finite approach, such as lower cost and better adherence to treatment, are taken into consideration.

The duration of any NUC consolidation therapy after achieving the criterion for cessation of treatment is another issue that must be addressed when optimizing the finite therapy approach [6, 7]. Previous guidelines have suggested the use of 6–12 months of NUC consolidation therapy after HBeAg seroconversion [1–3], but there is no evidence-based suggestion for discontinuation of finite therapy after the loss of HBsAg. In the present study, long-term consolidation with NUCs (>1 year) did not improve patient outcomes compared with short-term consolidation (<1 year). Notably, 9 (60%) of the patients in the finite NUC group received no consolidation therapy at all, suggesting that elimination of NUC therapy when HBsAg levels fall below 0.05 IU/mL could be an acceptable choice.

A number of laboratory methods and brands are available to measure HBsAg, and there is variability among them [13]. Therefore, additional research is needed to assess whether these various techniques are sufficiently similar to each other or whether standardization of the methodology is required.

The optimal experimental design to identify the endpoint of finite NUC therapy would be a randomized clinical trial. However, the potential endpoints currently under study do not occur frequently and are hard to predict, making a randomized clinical trial an impractical and uneconomical study design. For this reason, cohort studies and retrospective analyses make up the majority of completed studies in this field. Other limitations of this study also have to be considered. The sample size was small because of the rarity of loss of HBsAg, and the patients were from a single center. In addition, it was not possible to analyze some markers because their data were not included in the original database.

## 5. Conclusions

In conclusion, discontinuation of NUC therapy in patients with CHB could be acceptable in those in whom the HBsAg level falls to <0.05 IU/mL. Furthermore, consolidation therapy lasting <1 year could be adequate for the prevention of a poor long-term prognosis.

## Figures and Tables

**Figure 1:** Patient enrolment. HBsAg: hepatitis B surface antigen; HCC: hepatocellular carcinoma; NUCs: nucleos(t)ide analogues.

**Figure 2:** Long-term outcomes of patients with chronic hepatitis B given finite or indefinite NUC therapy after HBsAg had reached <0.05 IU/mL. ^∗^*P* < 0.05, ^∗∗^*P* < 0.01, and ^∗∗∗^*P* < 0.001. ALT: alanine aminotransferase; HBsAg: hepatitis B surface antigen; NUCs: nucleos(t)ide analogues.

**Figure 3:** Long-term outcomes of patients with chronic hepatitis B given finite NUC therapy that was withdrawn when HBsAg reached <0.05 IU/mL or indefinite NUC therapy after HBsAg reached <0.05 IU/mL. ^∗^*P* < 0.05. ALT: alanine aminotransferase; HBsAg: hepatitis B surface antigen; NUCs: nucleos(t)ide analogues.

**Figure 4:** Distribution of the duration of NUC consolidation therapy after HBsAg had fallen to <0.05 IU/mL in the finite NUC group. NUCs: nucleos(t)ide analogues; HBsAg: hepatitis B surface antigen.

**Figure 5:** Long-term outcomes of patients with chronic hepatitis B given long-term or short-term consolidation therapy with NUCs after HBsAg had reached <0.05 IU/mL. ALT: alanine aminotransferase; HBsAg: hepatitis B surface antigen; NUCs: nucleos(t)ide analogues.

**Figure 6:** Long-term outcomes of patients with chronic hepatitis B after withdrawal of long-term or short-term consolidation therapy with NUCs. ALT: alanine aminotransferase; HBsAg: hepatitis B surface antigen; NUCs: nucleos(t)ide analogues.

**Table 1:** Demographic and clinical characteristics of the patients.

Characteristic	Indefinite NUC group (*n* = 40)	Finite NUC group (*n* = 31)	*P*
Gender			0.999
Male	34 (85.0%)	27 (87.1%)	
Female	6 (15.0%)	4 (12.9%)	
Fatty liver	12 (30.0%)	10 (32.3%)	0.999
Initial NUC used			0.316
Lamivudine	11 (27.5%)	12 (38.7%)	
Entecavir	11 (27.5%)	9 (29.0%)	
Telbivudine	14 (35.0%)	5 (16.1%)	
Adefovir	4 (10.0%)	5 (16.1%)	
At start of NUC therapy			
Age (years)	41.2 (27.3–78.9)	38.9 (19.67–61.84)	0.397
HBeAg-positive	19 (47.5%)	16 (51.6%)	0.917
HBV DNA (copies/mL)	3.86 × 10^5^ (4.90 × 10^2^–6.82 × 10^7^)	1.52 × 10^6^ (1.00 × 10^3^–4.6 × 10^8^)	0.059
ALT (U/L)	113 (7–2293)	85 (21–752)	0.664
Albumin (g/L)	44 (30.1–49)	45.0 (35.8–51.8)	0.128
Total bilirubin (*μ*mol/L)	15.39 (4.7–75.4)	17.9 (5.4–45.9)	0.423
At HBsAg reaching <0.05 IU/mL			
Age (years)	45.8 (29.4–79.4)	47.4 (28.1–65.5)	0.531
Time for HBsAg to reach <0.05 IU/mL (weeks)	240 (1–672)	192 (12–480)	0.848
ALT (U/L)	29.5 (12–84)	24 (13–65)	0.407
Albumin (g/L)	45.9 (31.9–53)	47 (31.5–50.1)	0.118
Total bilirubin (*μ*mol/L)	12.8 (5.7–28.9)	14.4 (7.3–42.5)	0.958

Data are presented as *n* (%) or median (range). ALT: alanine aminotransferase; HBeAg: Hepatitis B e antigen; HBsAg: hepatitis B surface antigen; HBV: hepatitis B virus; NUC: nucleos(t)ide analogue.

**Table 2:** Characteristics of the patients in the finite NUC group at the time when HBsAg reached <0.05 IU/mL and the time when NUC therapy was withdrawn.

Characteristic	NUC withdrawal	HBsAg < 0.05 IU/mL	*P*
Age (years)	47.4 (28.1–65.5)	44.9 (25.7–65.5)	0.668
ALT (U/L)	24 (13–65)	27.5 (13–106)	0.756
Albumin (g/L)	47 (31.5–50.1)	46.9 (32.5–49.9)	0.822
Total bilirubin (*μ*mol/L)	14.4 (7.3–42.5)	13.7 (5.6–48.0)	0.927

**Table 3:** Characteristics of the patients in the finite NUC group with short-term (<1 year) or long-term (≥1 year) consolidation therapy with NUCs.

Characteristic	Short-term NUC consolidation (*n* = 15)	Long-term NUC consolidation (*n* = 16)	*P*
Gender			0.043
Male	11 (73.3%)	0 (0.0%)	
Female	4 (26.7%)	16 (100.0%)	
Fatty liver	3 (20.0%)	7 (43.8%)	0.252
Initial NUC used			0.491
Lamivudine	7 (46.7%)	5 (31.2%)	
Entecavir	4 (26.7%)	5 (31.2%)	
Telbivudine	1 (6.7%)	4 (25.0%)	
Adefovir	3 (20.0%)	2 (12.5%)	
At start of NUC therapy			
Age (years)	43.7 (23.3–61.8)	36.5 (19.7–60.1)	0.247
HBeAg-positive	6 (40.0%)	10 (62.5%)	0.372
HBV DNA (copies/mL)	5.84 × 10^5^ (1.00 × 10^3^–1.00 × 10^8^)	3.77 × 10^6^ (1.00 × 10^3^–4.60 × 10^8^)	0.101
ALT (U/L)	76 (21–752)	91 (25–752)	0.470
Albumin (g/L)	45 (40.8–51.8)	44.2 (35.8–49.7)	0.281
Total bilirubin (*μ*mol/L)	20.5 (9.6–45.9)	15.8 (5.4–39.5)	0.188
At HBsAg reaching <0.05 IU/mL			
Age (years)	48.2 (32.6–65.5)	41.0 (28.1–65.1)	0.323
Time for HBsAg to reach <0.05 IU/mL (weeks)	192 (12–480)	192 (60–408)	0.705
ALT (U/L)	21 (13–51)	28 (14–65)	0.066
Albumin (g/L)	47.0 (42.7–49.9)	47.4 (31.5–50.1)	0.843
Total bilirubin (*μ*mol/L)	14.8 (7.3–26.7)	13.7 (7.5–42.5)	0.812
At withdraw of NUCs			
Age (years)	48.2 (32.6–65.5)	39.7 (25.7–62.9)	0.167
ALT (U/L)	21 (13–106)	35 (17–73)	0.050
Albumin (g/L)	47 (42.7–49.9)	46.6 (32.5–49.7)	0.874
Total bilirubin (*μ*mol/L)	14.2 (7.5–26.7)	12.7 (5.6–48.0)	0.678

Data are presented as *n* (%) or median (range). ALT: alanine aminotransferase; HBeAg: Hepatitis B e antigen; HBsAg: hepatitis B surface antigen; HBV: hepatitis B virus; NUC: nucleos(t)ide analogue.

## Data Availability

The data set supporting the results of this article is included within the article.

## Supplementary Materials

Supplementary Materials Two statistical databases (PDF) of this study have been placed in supplementary files.
